The article "Enhancement of Patient Facial Recognition through Deep Learning Algorithm: ConvNet" was published in 2021. Journal: J Healthc Eng.

# Enhancement of Patient Facial Recognition through Deep Learning Algorithm: ConvNet

**DOI:** 10.1155/2021/5196000

**Published:** 2021-12-06

**Authors:** Edeh Michael Onyema, Piyush Kumar Shukla, Surjeet Dalal, Mayuri Neeraj Mathur, Mohammed Zakariah, Basant Tiwari

**Affiliations:** ^1^Department of Mathematics and Computer Science, Coal City University, Enugu, Nigeria; ^2^Computer Science & Engineering Department, University Institute of Technology, Rajiv Gandhi Proudyogiki Vishwavidyalaya, Bhopal 462033, India; ^3^College of Computing Science & IT, Teerthanker Mahaveer University, Moradabad, U.P.244001, India; ^4^SRM University, Delhi-NCR, Sonipat, Haryana 131039, India; ^5^College of Computer and Information Sciences, King Saud University, Riyadh, Saudi Arabia; ^6^Hawassa University, Awasa, Ethiopia

## Abstract

The use of machine learning algorithms for facial expression recognition and patient monitoring is a growing area of research interest. In this study, we present a technique for facial expression recognition based on deep learning algorithm: convolutional neural network (ConvNet). Data were collected from the FER2013 dataset that contains samples of seven universal facial expressions for training. The results show that the presented technique improves facial expression recognition accuracy without encoding several layers of CNN that lead to a computationally costly model. This study proffers solutions to the issues of high computational cost due to the implementation of facial expression recognition by providing a model close to the accuracy of the state-of-the-art model. The study concludes that deep l\earning-enabled facial expression recognition techniques enhance accuracy, better facial recognition, and interpretation of facial expressions and features that promote efficiency and prediction in the health sector.

## 1. Introduction

Facial expression is a nonverbal way of communication among humans. Facial expressions are representation of the emotional state of a human and have a huge impact on conveying emotions. The technique of recognizing a person's facial expression category is known as facial expression recognition. Facial expression recognition is utilized in a variety of applications, including the identification of mental disorders, depression analysis, and health forecasting and criminal detection. The seven universal facial expressions that are recognized in humans are “Happy, Sad, Fear, Anger, Surprise, Disgust, and Neutral.” This study focused on the classification of aforementioned facial expression with the help of deep learning techniques. In recent time, several techniques have been devised for automatic facial expression recognition with the help of deep neural networks. Deep neural networks are the subfield of machine learning that involve neural networks for figuring out solutions for the problems dealing with artificial intelligence [1]. Deep neural networks replicate the neocortex of the human brain that has several neurons. These neurons are used to build the neural network in deep learning models. Deep learning has various types of neural network models [2–4].

Convolutional neural networks (CNN/ConvNet) are used for application based on image classification, object detection, image processing, and so on. ConvNet has several layers and each layer has a different purpose. The layers in a CNN are input layer, convolutional layer, detector layer, pooling layer, and output layer. The input layer of ConvNet is the layer in which the input, for instance, an image, is given. This image is converted into discrete values of pixels corresponding to the coordinates of an image. The output of this layer is passed to the detector layer to convert linear data into a nonlinear data with the help of rectilinear activation. The feature map of this layer is passed as purpose of providing input to the pooling layer. This layer is utilized for the dimensionality reduction of the feature map and enables invariance upon small translations on the input. These layers comprise the basic architecture of convolutional neural networks [5–8].

Since CNNs help in 2D representation of an image, one can leverage this feature of CNN to locate positions of features of the input image and further can implement required translation on the images for the purpose of image processing. Modification in traditional architecture of convolutional neural network leads to better solutions of several problems that could not be catered by existing traditional models. Some of the architectures that are designed using traditional CNN models are LeNet, AlexNet, and GoogleNet [9]. These architectures are the result of modifications done in the traditional model of CNN by increasing or decreasing the number of layers used in convolutional neural networks. For the MNIST dataset, LeNet has an input layer of 32 × 32 pixels, a first convolution layer of 28 × 28 pixels, a pooling layer of 14 × 14 pixels, a second convolution layer of 10 × 10 pixels, a second pooling layer of 5 × 5, a third convolution of 1 × 1, a fully connected layer of 84 pixels, and a second fully connected (output) layer of 10 pixels [10–13]. AlexNet was made up of eight layers: five convolutional layers, three fully linked layers, and a ReLU activation function. The GoogleNet architecture employs a 1 × 1 convolutional layer and a global average pooling strategy to increase the neural network's depth capability. It includes an inception module [14] in addition to the CNN's basic design. At the input of the inception module, 1 × 1, 3 × 3, and 5 × 5 convolution, and 3 × 3 max pooling are all run in parallel, and the outputs are merged as the final output.

The researchers in this study employed ResNets to automatically classify facial expressions using the fer2013 dataset [15–17]. Facial expression provides a wealth of hidden information that can aid in the comprehension of human emotions and intentions and has a significant research value. We provide a strategy for facial expression recognition based on deep learning and CNN to overcome difficulties that commonly occur, such as low recognition accuracy and weak generalisation capacity of traditional face expression recognition algorithms. This method demonstrates the CNN model's capacity to recognise patient facial expressions more accurately.

## 2. Related Works

Hussain and Al Balushi [8] proposed the use of inception layers made up of 1 × 1, 3 × 3, and 5 × 5 convolution layers using ReLU activation function in parallel along with two convolution layers for the neural network model. While training the polynomial learning rate was considered as baselr (1 iter/maxiter) 0.5. Their model gave an accuracy of 0.693.

Suryanarayana et al. [18] explored the concept of the model based on Hist-eq technique which comprises of the first layer operated as the input transform and three layers operated as the convolutional and pooling layers, monitored by a fully connected two-layer MLP, and produced the most consistent results of all the network models. This model gave an accuracy of 0.6667.

Zhang et al. [11] proposed a cross-dataset approach for facial expression recognition in FER2013 dataset. Along with FER2013, they included three more datasets AFLW, Celeb-Faces, and Kaggle. These datasets have corresponding labels of the face attributes. They designed a bridging layer in order to use the features of these datasets unanimously and combine the output with FER2013 dataset. Their approach of facial expression recognition gave an accuracy of 0.71.

Devries et al. [16] developed a method for estimating the position and shape of facial landmarks, which aids in the improvement of facial expression identification. Their models include three completely connected convolutional layers, a fully connected ReLU hidden layer, and an output that uses the L2SVM activation function. They used data augmentation techniques such as mirroring, rotating, zooming, and rearranging the input photos at random. Their approach gave an accuracy of 0.6721. All the results have been shown in Table 1.

Khan et al. [9] stated that facial recognition is important for biometric authentication, which is utilized in a variety of applications, including security. To accomplish this goal, image processing techniques are used to change a stored database of the individuals. This study presents a smart glass architecture having capabilities of recognizing faces. Using portable smart glasses to implement facial recognition can help law enforcement authorities recognise a suspect's face. Their portability and superior frontal view capturing give them an edge over security cameras.

Mollahosseini et al. [19] presented that machine learning techniques were used throughout the face recognition process due to their high accuracy when compared to other techniques. Face detection, which uses Haar-like features, is the first step in face recognition [20]. Using 3099 features, this technique has a detection rate of 98 percent. Convolutional neural networks [21], a subfield of deep learning, are used to recognise faces (CNN). It is a multilayer network that uses categorization to do a certain task. For facial recognition, transfer learning of a trained CNN model called AlexNet is used. With 2500 variation photos in a class, it has a 98.5 percent accuracy rate [22]. These smart glasses can be used in the authentication procedure in the security area.

Fabian Benitez-Quiroz et al. [17] introduced a dynamic facial expression recognition (FER) method based on a two-stream architecture with both spatial and temporal CNN with local binary patterns on three orthogonal plane (LBP-TOP) feature in their paper. The suggested approach focuses on geographical features with obvious expression frames, as well as temporal information in all expression sequences that have been changed from nonexpression frames [23]. By tracking the optical flow information on the temporal part, this two-stream architecture has been proven in the field of action identification in video.

Zhang et al. [24] presented ways to apply LBP-TOP feature to extract the spatial-temporal feature on the process of facial expression change, and its effectiveness was proven in this sector. CK+ is used to test the proposed approach. And the results are equivalent to cutting-edge methodologies for demonstrating the efficacy of proposed architecture.

Storey et al. [25] presented details of the EmotioNet challenge approach and results in [11]. This is the first task to put computer vision algorithms [26] to the test in terms of automatically analyzing a huge number of photos of facial expressions of emotion in the wild. The task was split into two sections. The first track assessed the ability of existing computer vision techniques to detect action units automatically (AUs). We examined the detection of 11 AUs in particular. The computers' capacity to distinguish emotion categories [20] in photographs of facial expressions was tested in the second track.

Wang et al. [27] investigated the recognition of 16 basic and compound emotion types in particular. The challenge's results indicate that current computer vision and machine learning algorithms are unable to accomplish these two objectives reliably. When attempting to discern emotion, the limits of present algorithms [22] become more evident.

Georgescu et al. [28] show that minor resolution modifications, small occludes, gender, or age have no effect on present algorithms, but that 3D posture is a substantial performance limiting issue. We go over the areas that need to be addressed more closely moving forward in detail.

Alelaiwi [29] discussed that smart healthcare systems are more accurate and dependable when they incorporate multimodal inputs. It is proposed in this paper to use a multimodal input system made of users' facial images and speech to assess their happiness. All of the inputs are processed, and the findings are distributed to various stakeholders in the smart healthcare environment based on their level of satisfaction. During cloud processing, a slew of image [30] and voice features are extracted. Speech and picture features are represented using directional derivatives and a weber local descriptor, respectively. Using support vector machines, the features are integrated into a multimodal signal and fed to a classifier. The proposed technique has a satisfaction detection accuracy of 93%. Experiments show the proposed multimodal HR sensor outperforms existing single-modal HR sensors based primarily on rPPG or BCG in terms of robustness and accuracy. Ten patients had a 100% success rate in identifying their emotions based on their relaxed and tense facial expressions. Each patient's motion prediction accuracy was compared to the accuracy [31] of the observed emotions using a heatmap.

Muhammad et al. [32] proposed healthcare framework that uses a facial expression recognition system which may benefit from the fact that human facial expressions fluctuate as one's health changes. A large amount of data is used in several experiments to verify the proposed system. At least 99.95% of the proposed system's experimental results show it can accurately recognise facial expressions.

Pikulkaew et al. [33] stated that there will always be pain; therefore, this study looks at how facial expression technology can help those who are suffering from it. We have a process that may classify pain as not painful, painful, or painfully painful. An expert physician's conclusions were compared to the system's to assess the system's overall performance. Classification precision rates were 99.75% for not painful, 92.93% for painfully becoming painful, and 95.15% for painfully being painful. To summarize, our research has produced a simple, cost-effective, and simply understood alternate technique for the general public and healthcare [34] professionals to screen for pain prior to admission. This sort of analysis could also be used to discover infectious diseases through the use of pain.

Previous research [35, 36] shows that deep learning has delivered breakthrough outcomes in numerous application sectors, including speech recognition and picture recognition, over the last few years. With other things, we are attempting to use deep learning algorithms [37] to detect real-time facial expressions. Instead of relying on handcrafted feature-based techniques, the proposed system is capable of recognizing using a webcam and creates human emotions based on face expressions [38]. It can distinguish and detect faces.

## 3. Methodology

In this section, we will discuss the models and methodologies used by us for facial expression recognition. There are different data augmentations applied to FER2013 dataset in order to increase the samples in the dataset. Along with data augmentation, we have designed the convolutional neural network model by introducing a residual block in the existing ConvNet model. We have chosen different sets of parameters for optimizing the model and to improve the learning of the model. The methodology used in this study is depicted in Figure 1.

### 3.1. Data Augmentation

The purpose of the data augmentation is to resolve the issue of limited samples in the dataset to some extent along with increasing the diversity of the data. Commonly used data augmentations are flip, rotation, scale, crop, translation, and Gaussian noise along with some advanced data augmentation techniques. In this paper, we have used data augmentation technique that randomly crops the image into 4 parts along with the center crop and each cropped image is padded with the mirror of the cropped image. We have also applied random flip data augmentation technique [19, 24, 39–41].

### 3.2. Neural Network Model

The convolutional neural network [42] model implemented in our work is ResNets. The basic architecture of ResNets is shown in Figure 2. ResNets are used for dealing with the issue of vanishing/exploding gradient when increasing the number of layers in the model which leads to large error values at the time of training and testing [43]. Residual block uses a technique of skip connections which skips few layers in the neural network and connects directly to the output [18, 27, 29, 44]. The advantage of using ResNets is that it reduces the computational cost of processing the information in several layers by skipping the few layers in neural network leading to a model with few layers as compared to the existing models used [32, 45–48]. In our model, we have a pooling layer, two convolution layers each of 64 × 64, a first ResNet block using the output of the second convolutional layer and a 512 × 512 convolutional block using the output of the third. We also have a third convolutional layer of 128 × 128 and another pooling layer and a fourth convolutional layer of 512 with a pooling layer. We have used rectilinear activation function in our model. We also included the concept of batch normalization in our model in order to reduce internal covariance and instability in order to avoid overfitting.

Parameters used: to calculate the loss generated at the time of training the model we have incorporated the cross-entropy loss as our loss function. To optimize the loss generated during training the model, we have implemented in the Adam optimizer. The proposed approach has used one-cycle learning scheduler with the maximum learning rate of 0.001. We trained the model using these parameters for maximum 40 epochs. With these parameters, we could attain the maximum accuracy of our model on FER2013 dataset.

### 3.3. Data

There are several datasets that exist for the facial expression recognition systems. Few most commonly used datasets are mentioned below.

- CK+
- MMI
- JAFFE
- FER2013

Figure 3 shows the samples from the FER2013 dataset that were automatically gathered using Google's Image Search API. This is a train set, a validation set, and a test train set, all with a combined total of 23,000 photos. Each image belongs to a class that is labelled as the seven universal expressions, “Happy, Sad, Anger, Disgust, Fear, Neutral, and Surprise.” There are total of 35,887 images that are grayscale and 48 × 48 pixels in size. Image 3 displays a selection of photographs from the dataset. The deep learning model for facial expression identification was trained on FER 2013 dataset.

## 4. Result and Discussion

In this section, we will mention the results deduced on implementation of the methods mentioned in the proposed work.  Figure 4 shows the confusion matrix that includes the accuracies per class as well as overall accuracy on FER2013 dataset. As shown in the confusion matrix, our model attained an accuracy of 0.70 which is very close to the state-of-the-art model that already exists but just with a fewer number of layers.  Figure 5 shows accuracy on the test set after training the model.

A combination of ResNets and standard convolutional neural networks was used for facial expression identification on the FER2013 dataset, as illustrated in Figure 5.

As indicated by Figure 6, our model (result) gave an accuracy of 0.70 after reducing the number of layers in our convolutional neural network [20] leading to a computationally cheaper model as compared to the existing models that require several layers for classification in convolutional neural networks.  Figure 7 demonstrated the cycle learning rate with respect to batch nos.

This accuracy level of the proposed model plays very good role in the patient monitoring situations and prediction of their activities through their facial expression. The technique presented in this study would assist physicians to improve their services and also the computer to make accurate health predictions [22].

## 5. Discussion

Facial expressions offer a wealth of nonverbal information that can be used in the study to better comprehend human emotions and intentions. The approach we presented in this study proved effective in patient facial expression recognition performance and provided a new way to solve problems in the existing ones as presented earlier in the literature. Our new approach enables face expression to be recognized and classified effectively with more accurate thereby reducing the computational cost and time consumption and improving the image recognition rate. The model is developed to improve the accuracy of patient face image classification. Our result shows that deep learning-enabled facial expression recognition technique enhances accuracy, better facial recognition, and interpretation of facial expressions and features that would promote efficiency [49] and prediction in the health sector.

## 6. Conclusion

Facial expression emotion identification is a fascinating area of the study that has been applied in a variety of contexts, including safety, health, and human-machine interfaces. Researchers in this area are working to improve computer predictions by developing ways for interpreting, coding, and extracting facial expressions. Because of deep learning's exceptional success, several sorts of architectures are being used to improve performance.

Since our presented model is computationally cheaper, it can be incorporated with other models in order to improve the accuracy of facial recognition systems using FER2013 dataset. Though FER2013 dataset is a very complex dataset with a limited number of samples per class, in order to improve the accuracy, the number of samples in each class can be increased by an optimal amount. Facial expression recognition can be combined with the concept of natural language processing (NLP) in order to increase the dimensionality of automatic facial expression recognition systems. If the future scope is implemented, it can play more important roles in e-Health system and health service delivery.

## Figures and Tables

**Figure 1:** Proposed methodology.

**Figure 2:** ResNet.

**Figure 3:** FER2013 dataset (kaggle.com/msambare/fer2013).

**Figure 4:** Confusion matrix.

**Figure 5:** Accuracy.

**Figure 6:** Loss vs. epoch.

**Figure 7:** One-cycle learning rate.

**Table 1:** Existing work analysis.

Model	Accuracy
Mollahosseini et al. [19]	0.693
Feng and Ren [13]	0.6667
Zhang et al. [11]	0.71
Devries et al. [16]	0.6721

## Data Availability

The data that support the findings of this study are available upon request from the corresponding author.
